RETRACTED

# Effect of Supplementation of Vitamin D in Patients with Periodontitis Evaluated before and after Nonsurgical Therapy

**DOI:** 10.1155/2022/5869676

**Published:** 2022-08-08

**Authors:** Shree Mohan Mishra, P. L. Ravishankar, V. Pramod, Prem Blaisie Rajula, K. Gayathri, Mohammad Khursheed Alam, A. Thirumal Raj, Shilpa Bhandi, Shankargouda Patil

**Affiliations:** ^1^Department of Periodontology, New Horizon Dental College, Bilaspur, 495001 Chattisgarh, India; ^2^Department of Periodontology, SRM Kattankulathur Dental College & Hospital, SRM lnstitute of Science and Technology, SRM Nagar, Kattankulathur, 603203 Kancheepuram, Chennai, Tamil Nadu, India; ^3^Orthodontics, Preventive Dentistry Department, College of Dentistry, Jouf University, Sakaka 72345, Saudi Arabia; ^4^Center for Transdisciplinary Research (CFTR), Saveetha Dental College, Saveetha Institute of Medical and Technical Sciences, Saveetha University, Chennai, India; ^5^Department of Public Health, Faculty of Allied Health Sciences, Daffodil lnternational University, Dhaka, Bangladesh; ^6^Department of Oral Pathology and Microbiology, Sri Venkateswara Dental College and Hospital, Chennai 600130, India; ^7^Department of Restorative Dental Sciences, Division of Operative Dentistry, College of Dentistry, Jazan University, Jazan 45142, Saudi Arabia; ^8^Department of Cariology, Saveetha Dental College & Hospitals, Saveetha Institute of Medical and Technical Sciences, Saveetha University, Chennai- 600 077, India; ^9^Department of Maxillofacial Surgery and Diagnostic Science, Division of Oral Pathology, College of Dentistry, Jazan University, Jazan 45142, Jazan 45412, Saudi Arabia; ^10^Centre of Molecular Medicine and Diagnostics (COMManD), Saveetha Dental College & Hospitals, Saveetha Institute of Medical and Technical Sciences, Saveetha University, Chennai- 600 077, India

## Abstract

**Background:**

Vitamin D has anti-inflammatory properties and the potential to increase the generation of antimicrobial peptides like cathelicidin and defensins that may have a good impact on oral health. Higher vitamin D consumption has also been linked to a reduced risk of periodontal disease progression. Hence, the primary objective of this study was to evaluate and compare the clinical and laboratory parameters of oral supplementation of vitamin D as an adjuvant to scaling and root planing and to assess the bone mineral density via qualitative ultrasound bone density scanner in chronic periodontitis patients. *Methodology*. This study included 40 patients with periodontitis categorized into 2 groups with twenty patients each, Group I comprising scaling and root planing (SRP) alone and Group II comprising SRP along with vitamin D supplementation. Plaque index, gingival index, probing pocket depth, and clinical attachment loss was measured as clinical parameters. Serum vitamin D levels were assessed before and after SRP at both baseline and 6 weeks.

RETRACTED

**Results:**

The intergroup comparison of clinical parameters (PI, GI, PPD, and CAL) at 6 weeks for both the groups showed statistical significance. Intragroup comparison of clinical parameters from baseline to 6 weeks showed a statistically significant reduction in both groups. The mean bone mineral density level in both the control and test groups demonstrated a mean *T* score of –1.3 and –1.21, respectively. The mean vitamin D levels were 27.8460 and 28.1020 for the test and control groups, respectively, which was statistically insignificant (*p* = 0.705) and those at six-week intervals improved to 31.3650 and 28.0240 which were statistically significant (*p* ≤ 0.001).

**Conclusion:**

It could be stated that a positive relationship exists between periodontitis and osteopenia which could aggravate periodontal destruction. All periodontitis cases should thus be evaluated for BMD and supplemented with vitamin D_3_ in an appropriate dosage and time frame to treat both these diseases.

## 1. Introduction

The most common type of periodontitis is periodontitis, which is characterized by a slow progression of inflammatory disease. Systemic and environmental variables (e.g., diabetes, smoking) may change the host's immunological response to the tooth biofilm, causing periodontal damage to occur more quickly [1]. Inflammatory and immune reactions that extend deep into the connective tissue beyond the cementoenamel junction (CEJ) may include loss of connective tissue attachment to the tooth involved as well as loss of the alveolar bone.

Alveolar bone loss is more common in people with osteoporosis or low bone mass, according to research, though this connection is not fully accepted. A negative calcium balance is likely to come from a chronically low intake of vitamin D and calcium, leading to an increase in calcium removal from bone, including the alveolar bone. The tooth attachment system may be weakened as a result of this bone loss.

Vitamin D, namely, 1,25-dihydroxy vitamin D, has anti-inflammatory and antimicrobial properties via modifying immune cell cytokine production and increasing monocyte-macrophage cell secretion of antibacterial peptides. Vitamin D's various functions could help people with periodontal disease.

The inflammatory response, which is triggered by endotoxins or by the stimulation of the host immune system and the production of inflammatory mediators, causes tissue destruction. By initiating osteoclast-mediated bone resorption, these locally generated compounds cause connective tissue degradation and bone loss [2].

RETRACTED

The general population's vitamin D and calcium intake should be within current limitations of 400 to 600 IU and 1,000 to 1,200 mg daily, respectively. Despite a growing agreement that such routine limits are insufficient, and professional organizations now prescribe increased vitamin D dosages (800 to 1,000 IU daily), 1 billion people are believed to be vitamin D deficient or insufficient globally. Although many people are aware of the benefits of calcium and vitamin D supplementation for bone health, their role in periodontal disease remains unknown. Taking vitamin D and/or calcium has been shown to prevent alveolar bone breakdown, gingivitis, and attachment loss in several trials [3].

Vitamin D is a potent anti-inflammatory and antimicrobial agent. Vitamin D is also required for bone strength and calcification, which appears to include alveolar bone. It was also recently reported that a higher vitamin D intake may protect against periodontal disease progression in older men. On the other side, no correlation exists between vitamin D levels and radiographic assessments of alveolar crest height (ACH), which are assumed to characterize the chronic stage of damaging periodontitis. Few studies have looked at the relationship between periodontal disease markers and vitamin D levels throughout time [4]. The goal of this study will be whether using vitamin D oral supplementation as an addition to periodontal treatment improves clinical measures of periodontal health.

## 2. Methodology

The present study was approved by the institutional ethics committee of New Horizon Dental College and Research Institute (ref. no NHDC&RI/2014/8340). Informed consent was obtained from all the patients.

The present randomized case-control clinical study comprising 40 patients with periodontitis was designed and implemented in the Department of Periodontology, New Horizon Dental College and Research Institute, Sakri, Bilaspur, Chhattisgarh. Systemically healthy patients within the age group of 19-50 years with generalized moderate to severe periodontitis (stage III) having a minimum of 20 teeth exhibiting probing depth ≥ 5 mm and CAL ≥ 5 mm were included in the study. Participants who underwent periodontal therapy, in the last 6 months, medically compromised patients (diabetes, hypertension, and CVS), osteoporosis, and patients with a history of disease, disorders, or drugs that might affect mineral metabolism and periodontal health are excluded. A detailed case history was recorded in a designed pro forma for all the patients, and written consent was obtained.

RETRACTED

### 2.1. Assessment of Parameters

Plaque index, gingival index, probing pocket depth, and clinical attachment loss was recorded as clinical parameters to assess periodontal condition before and after the intervention. After the clinical examination and biochemical evaluation (blood test), detailed case sheet documentation including medical history was carried out by a single calibrated examiner. Patients who had generalized CP were provisionally recruited into the study and categorized into two groups as follows:

- Group I (control): 20 subjects with periodontitis were subjected to SRP alone. Clinical parameters, bone mineral density, and serum vitamin D levels, were measured at baseline and six weeks after SRP
- Group II (test): consisting of 20 subjects with periodontitis were administered vitamin D supplements (Medisys® D_3_) (400 IU)/day for 6 weeks as an adjunct to SRP. Clinical parameters, bone mineral density and serum levels of vitamin D, were assessed at baseline and 6 weeks after SRP

Patients of both the groups were put on SRP, patient education, and motivation, and oral hygiene instructions were given.

### 2.2. Measurement of Vitamin D Levels and Bone Mineral Density

Serum vitamin D levels were assessed using the Chemiluminescent immune assay (ADVIA CENTAUR) (Thyrocare) technique at baseline and six weeks after therapy in both groups. Luminescent immunoassays are variations of the standard ELISA, just like fluorescent immunoassays. An enzyme converts a substrate to a reaction product that emits photons of light instead of developing a visible color.

Bone mineral density was measured by quantitative ultrasonography (QUS) using a bone mineral density scanner (Sunlight Ultrasound Bone Density Scanner). QUS is a noninvasive approach to determining bone mineral conditions in the periphery bone that is relatively new. QUS methods offer biomechanical information in addition to bone density, which may be useful in assessing fracture risk. The BMD using QUS was assessed in the radial bone and patients were categorized with a *T* score of normal: 0 to -1, osteopenia: -1 to -2.5, and osteoporotic: -2.5 and above. In patients, the density of the maxillary alveolar process bone is linked to the density of the mandibular alveolar ridge, vertebral column, hips, and radius [5].

### 2.3. Periodontal Intervention

Scaling and root planing (SRP) were performed by hand instruments (Gracey's Area Specific curettes from #1 to #14).

## 3. Statistical Analysis

The collected data were statistically analyzed. The standard deviation, standard error, and mean were determined. The Student *T*-test was used to determine the level of significance and the correlation of each treatment group's efficacy. All of the data was processed using the statistical program SPSS 15.0, and the findings were obtained using the student *T*-test. *p* value less than 0.05 was regarded as statistically significant (^∗^), and *p* value less than 0.001 was considered statistically highly significant (∗∗).

RETRACTED

## 4. Results

The present study included 40 generalized CP patients who were allocated under the two study groups. The intragroup comparison (Table 1) and intergroup comparison (Table 2) were done between the test and control groups at baseline and six weeks.

The mean plaque index values at baseline between the control and test groups were 1.55 and 1.652 which was statistically insignificant (*p* = 0.128) at the six-week interval reduced to 1.304 and 1.012 which were statistically highly significant (*p* ≤ 0.001), respectively. The mean gingival index values at baseline between the control and test groups were 1.560 and 1.517 which was statistically insignificant (*p* = 0.482) and those at six-week intervals reduced to 1.348 and 0.820 which were statistically highly significant (*p* ≤ 0.001), respectively. The mean probing pocket depth values at baseline between the control and test groups were 5.848 and 5.557 which was statistically insignificant (*p* = 0.301) and those at the six-week interval were reduced to 3.4702 and 2.7700 which were statistically significant (*p* = 0.037), respectively. The mean clinical attachment values at baseline between the control and test groups were 6.245 and 6.29 which was statistically insignificant (*p* = 0.869) and those at six-week intervals were reduced to 3.8200 and 2.9500 which were statistically significant (*p* = 0.035), respectively. The mean vitamin D levels were 27.8460 and 28.1020 for the test and control groups, respectively, which was statistically insignificant (*p* = 0.705) and those at six-week intervals improved to 31.3650 and 28.0240 which were statistically significant (*p* ≤ 0.001), respectively. The mean bone mineral density level values at baseline between the control and test groups were -1.3000 and -1.2100 which was statistically insignificant (*p* = 0.862) and those at six-week interval were -1.5450 and –1.3800 which was not significant (*p* = 0.456), respectively. The intragroup comparison of the clinical parameters from baseline to 6 weeks showed a statistically significant reduction in both the groups. The intergroup comparisons of the clinical parameters at baseline for both the groups were not statistically significant.

## 5. Discussion

Periodontitis is an inflammatory process of the teeth's surrounding tissues induced by a variety of microorganisms that causes progressive degradation of the periodontal ligament and alveolar bone loss, as well as increasing pocket depth, recession, or both [6].

RETRACTED

Persons with low bone mass or osteoporosis are more prone to alveolar bone loss. This type of bone loss can hasten the onset of periodontal disease [7]. Vitamin D deficiency affects almost every group of society, including children and young people. The Indian Council of Medical Research (ICMR) suggests consuming 400 IU of vitamin D each day [8]. 1,25-Dihydroxy vitamin (the active form of vitamin D) (vitamin D3) is a strong immunological modulator by inhibiting cytokine synthesis by immune cells and stimulating monocytes-macrophages to release antibiotic-active peptides [3].

Southard et al. did a study and concluded that vitamin D is used as a supplement in periodontal maintenance therapy, but very little research has been instituted on its use as an adjuvant to SRP [5]. Hence, this case-control study with 40 patients diagnosed with periodontitis was performed to see if there was a link between periodontitis and skeletal bone mineral density, as well as the effect of vitamin D supplementation combined with nonsurgical periodontal therapy.

The intragroup comparison of the clinical parameters from baseline to 6 weeks showed a statistical significant reduction in both the groups. The intergroup comparisons of the clinical parameters at baseline for both the groups were not statistically significant showing that cases with similar disease severity were recruited for the study.

The intergroup comparison of the clinical parameters (PI, GI, PPD, and CAL) at 6 weeks for both the groups showed statistically significant. This could be attributed to the decrease in gingival inflammation after the removal of local irritants following nonsurgical therapy. The significant decrease in the gingival index values in the test group at six-week intervals may attribute to the anti-inflammatory effects of vitamin D supplements (400 IU). This was in accordance with the study done by Hiremath et al. who found a dose-dependent anti-inflammatory effect of vitamin D supplementation on gingivitis patients [9].

A greater reduction of PPD from baseline to six weeks in both the groups could be attributed firstly to the beneficial effects of scaling and root planing on the soft tissues within the periodontal pocket leading to shrinkage and decrease in pocket depth. The superior result seen in the test group could be attributed to the positive effect of vitamin D on wound healing. The result of this study was in accordance with the previous study done by Tonguc et al. in which vitamin D administration improved healing potential [10].

RETRACTED

QUS is a simple, safe, and feasible technology. These are a compact instrument that takes just a few minutes to complete the measurements and emits minimal or zero radiation [11]. The mean bone mineral density level values at baseline between the control and test groups were -1.3000 and -1.2100 which was statistically insignificant (*p* = 0.862) and those at six-week interval were -1.5450 and -11.3800 which was nonsignificant (*p* = 0.456), respectively. The distinctive feature of this study was that the patients selected in both the control and test groups diagnosed with periodontitis demonstrated a mean *T* score of –1.3 and –1.21, respectively, which could be grouped as osteopenia patients. This exhibits a correlation between osteopenia and periodontitis and is in accordance with a study (Hattatoglu-Sonmez et al.) done previously [12]. Considering this dual relationship, it may be stated that all patients with periodontitis may be screened for their skeletal bone mineral density and treated appropriately as the bone of lesser density may be more prone to rapid destruction caused by periodontal infection [13].

Vitamin D supplementation elevated the bone mineral density in the test group at six weeks (-1.38) as compared to the control (-1.54) though the patients still remained in the osteopenia range. This could be because vitamin D suppresses OPG expression, and the combination of high RANKL expression and low OPG expression mediated by vitamin D would promote osteoclast differentiation and stimulation, as well as enhanced bone resorption [13]. Low vitamin D levels may also raise parathyroid hormone levels in the blood, which can promote bone resorption and elevate blood calcium levels indirectly.

In this study, vitamin D was administered only for six weeks which may have been an insufficient time interval to produce changes in bone mineral density. Thus, it could be stated that a positive relationship exists between periodontitis and osteopenia which could aggravate periodontal destruction. All periodontitis cases should thus be evaluated for BMD and be supplemented with vitamin D_3_ in an appropriate dosage and for an adequate time frame to treat both these chronic diseases appropriately [14].

## 6. Conclusion

In conclusion, the current study's findings revealed that there is a link between periodontitis and osteopenia. As a result, these individuals might be tested for bone mineral density and serum vitamin D levels. Vitamin D supplements can be utilized in conjunction with SRP to enhance periodontal disease status and bone mineral density.

## Figures and Tables

**Table 1:** Intragroup comparison of parameters at baseline and six weeks in the test and control groups.

Time interval	Control		Test	
Plaque index	Mean	*p* value	Mean	*p* value
Gingival index	0.152	0.018^∗^	0.246	*p* ≤ 0.001^∗∗^
Probing pocket depth	0.697	*p* ≤ 0.001^∗∗^	0.212	0.037^∗^
Clinical attachment level	2.787	*p* ≤ 0.001^∗∗^	2.377	*p* ≤ 0.001^∗∗^
Serum vitamin D	2.216	*p* ≤ 0.001^∗∗^	0.959	*p* ≤ 0.001^∗∗^
Bone mineral density	-3.519	*p* ≤ 0.001^∗∗^	0.078	0.236^∗^
Plaque index	0.17000	0.495	0.24500	0.349

^∗^Statistically significant. ^∗∗^Statistically highly significant.

RETRACTED

**Table 2:** Inter-group Comparison of Mean values at Baseline and at 6 weeks.

Parameters (mean)	Baseline		*p* value	6 weeks		*p* value
	Control	Test		Control	Test	
Plaque index	1.550	1.652	0.128	1.304	1.012	*p* ≤ 0.001^∗∗^
Gingival index	1.560	1.517	0.482	1.348	0.820	*p* ≤ 0.001^∗∗^
Probing pocket depth	5.848	5.557	0.301	3.470	2.770	*p* ≤ 0.001^∗∗^
Clinical attachment level	6.245	6.290	0.869	3.820	2.950	0.035^∗^
Serum vitamin D	28.102	27.846	0.705	28.024	31.365	*p* ≤ 0.001^∗∗^
Bone mineral density	-1.300	-1.210	0.862	-1.545	-1.380	0.456

^∗^Statistically significant. ^∗∗^Statistically highly significant.

## Data Availability

No data were used to support this study.
